The article "Bevacizumab-Induced Mitochondrial Dysfunction, Endoplasmic Reticulum Stress, and ERK Inactivation Contribute to Cardiotoxicity" was published in 2021. Journal: Oxid Med Cell Longev.

# Bevacizumab-Induced Mitochondrial Dysfunction, Endoplasmic Reticulum Stress, and ERK Inactivation Contribute to Cardiotoxicity

**DOI:** 10.1155/2021/5548130

**Published:** 2021-03-17

**Authors:** Yue Li, Wei Tian, Dongsheng Yue, Chen Chen, Chenguang Li, Zhenfa Zhang, Changli Wang

**Affiliations:** ^1^Department of Lung Cancer, Tianjin Medical University Cancer Institute and Hospital, National Clinical Research Center for Cancer, Key Laboratory of Cancer Prevention and Therapy, Tianjin's Clinical Research Center for Cancer, Tianjin Lung Cancer Center, Tianjin 300060, China; ^2^Department of General Surgery, The Second Affiliated Hospital of Tianjin University of Traditional Chinese Medicine, Tianjin 300060, China

## Abstract

The molecular mechanisms underlying the cardiotoxicity associated with bevacizumab, a first-line immunotherapeutic agent used to treat lung cancer, are not fully understood. Here, we examined intracellular signal transduction in cardiomyocytes after exposure to different doses of bevacizumab *in vitro*. Our results demonstrated that bevacizumab significantly and dose-dependently reduces cardiomyocyte viability and increases cell apoptosis. Bevacizumab treatment also led to mitochondrial dysfunction in cardiomyocytes, as evidenced by the decreased ATP production, increased ROS production, attenuated antioxidative enzyme levels, and reduced respiratory complex function. In addition, bevacizumab induced intracellular calcium overload, ER stress, and caspase-12 activation. Finally, bevacizumab treatment inhibited the ERK signaling pathway, which, in turn, significantly reduced cardiomyocyte viability and contributed to mitochondrial dysfunction. Together, our results demonstrate that bevacizumab-mediated cardiotoxicity is associated with mitochondrial dysfunction, ER stress, and ERK pathway inactivation. These findings may provide potential treatment targets to attenuate myocardial injury during lung cancer immunotherapy.

## 1. Introduction

Bevacizumab is a first-line immunotherapeutic agent used for the treatment of lung cancer [1]. The cancer-suppressing effects of bevacizumab are associated with inhibition of vascular endothelial growth factor signaling, which leads to decreased tumor growth and impaired invasion [2, 3]. However, bevacizumab is also associated with cardiovascular toxicities, including decreased left ventricular ejection fraction, vasculitis, hypertension, arrhythmias, vascular bed degeneration, and limited angiogenesis response [4–8]. Several mechanisms, including accumulation of toxic metabolites, cardiac microvascular vasospasm, and excessive activation of the renin-angiotensin system, might underlie the adverse effects of bevacizumab on the heart [4–7]. However, the intracellular molecular mechanisms underlying bevacizumab-associated cardiotoxicity are not fully understood.

At the molecular level, cardiomyocyte viability and function are greatly affected by mitochondrial performance [9, 10]. Mitochondria regulate cardiomyocyte contraction and relaxation by controlling ATP production [11, 12]. As the primary site of protein manufacturing, the endoplasmic reticulum (ER) controls protein synthesis, folding, and release [13, 14]. Previous studies have reported that targeted cancer therapies, such as doxorubicin [15], anthracycline [16], and cantharidin [17], can result in cardiovascular toxicities. The adverse effects of chemotherapy drugs may result from impaired mitochondrial function, increased oxidative stress [15, 18], increased mitochondria-proteasome interactions [19], impaired mitochondrial autophagy [20, 21], activation of mitochondrial inflammation signaling pathways such as NF-*κ*B [22], mitochondrial energy metabolic dysfunction [23], and mitochondrial apoptosis [24]. In addition, ER-mediated abnormalities in intracellular calcium signaling, protein misfolding as a result of ER stress, and ER-dependent cell apoptosis [25–27] can also contribute to cardiomyocyte damage during chemotherapy. Whether bevacizumab-mediated cardiovascular disorders are attributable to mitochondrial damage and/or ER stress remains to be determined.

The MAPK/ERK signaling pathway plays an important role in cardiomyocyte survival under stress conditions [28, 29]. Activated ERK attenuates oxidative stress in cardiomyocytes by promoting the transcription of antioxidative stress genes [30]. In addition, ERK alleviated chronic cardiac hypertrophy by improving mitochondrial metabolism [31]. As in cardiomyocytes, ERK promotes growth during tumor proliferation and invasion, and upregulation of the ERK pathway increased angiogenesis [32]. The ERK pathway also affects immune response in various tumors [33, 34]. In this study, we examined whether mitochondrial dysfunction, ER stress, and the ERK pathway are involved in bevacizumab-induced cardiotoxicity.

## 2. Materials and Methods

### 2.1. Cell Culture

H9C2 cell lines purchased from ATCC were grown in DMEM supplemented with 10% fetal bovine serum. The cells were maintained at 37°C and 5% carbon dioxide in a humidified environment. Cardiomyocytes were incubated with 0.1 or 5 mM bevacizumab as described in previous studies. Cardiomyocytes were also incubated with PD98059, an ERK pathway inhibitor, as described in previous reports to examine the influence of ERK inhibition on cardiomyocyte viability.

### 2.2. Cell Viability Assay

A total of 3000 treated cells per well were seeded in 96-well culture plates and incubated with or without bevacizumab for the indicated times; fresh media containing 50 *μ*l of CCK8 solution (5 mg/ml) (Dojindo Laboratories, Kumamoto, Japan) was then added followed by incubation at 37°C for 3 hours according to the manufacturer's protocol [35]. Absorbance was measured at 450 nm using an enzyme e-linked immunosorbent assay reader [36].

### 2.3. Mitochondrial ROS Detection

Cardiomyocytes were treated with bevacizumab and then washed with cold PBS three times. Then, 0.5 ng/ml MitoSOX Red mitochondrial superoxide indicator (Molecular Probes, USA) was added to the cardiomyocyte medium and incubated for 30 minutes in the dark. Cells were then washed with cold PBS three times [37]. Mitochondrial ROS production was observed under a confocal laser scanning microscope (LSM780; Carl Zeiss, Oberkochen, Germany, or TCS SP8; Leica, Wetzlar, Germany) and an Axio Zoom V16 stereo microscope (Carl Zeiss) [38].

### 2.4. Intracellular Calcium Content

Intracellular calcium measurements were performed as previously described with minor modifications [39]. Briefly, H9C2 cells were loaded with 5 *μ*M Fluo4-AM calcium probe for 30 minutes at 37°C [40]. Cells were then washed with PBS, and intracellular calcium was observed under a confocal laser scanning microscope (LSM780; Carl Zeiss, Oberkochen, Germany, or TCS SP8; Leica, Wetzlar, Germany) and an Axio Zoom V16 stereo microscope (Carl Zeiss) [41].

### 2.5. Immunofluorescence

For fluorescence microscopy-based detection of target proteins, 5 *μ*m thick cryosections were deparaffinized in xylene and rehydrated through graded ethanol [42]. Antigen retrieval was performed for 20 min at 95°C with 0.1% sodium citrate buffer (pH 6.0). After endogenous peroxidase activity was quenched with 3% H_2_O_2_·dH_2_O and nonspecific binding was blocked with 1% bovine serum albumin buffer, sections were incubated overnight at 4°C with primary antibodies using an Alexa 594 TSA Kit (Invitrogen) according to the manufacturer's instructions [43]. Stained sections were observed under a confocal laser scanning microscope (LSM780; Carl Zeiss, Oberkochen, Germany, or TCS SP8; Leica, Wetzlar, Germany) and an Axio Zoom V16 stereo microscope (Carl Zeiss) [44].

### 2.6. Detection of GSH, SOD, and GPX Activities

GSH, SOD, and GPX activities were detected using a Zymography Assay Kit (Applygen Technologies, China) according to the manufacturer's protocol [45]. GSH, SOD, and GPX were separated by SDS-PAGE. SDS was then extracted from the gel by incubating with Triton X-100 for 48 hours at 37°C. Finally, the gels were stained with Coomassie Brilliant Blue G250 and decolorized. A bright band against the blue background indicated the activity of targeted proteins. A Gel Image System (image master 1D analysis software, Pharmacia) was used to image the band [46].

### 2.7. Western Blot Analysis

Cell lysate was boiled in a sample buffer (62.5 mM Tris-HCl, pH 6.8, 2% sodium dodecyl sulfate, 20% glycerol, and 10% 2-mercaptoethanol), and protein concentration was determined using a Bradford protein assay kit (Thermo Fisher Scientific, Waltham, MA, USA) with bovine serum albumin as the standard [47]. Following protein transfer, the membrane was blocked with 5% skim milk in PBS Tween- (PBST-) 20 for 2 h at room temperature and then incubated overnight with antibodies at 4°C (the primary antibodies include Bcl2, 1 : 1000, Cell Signaling Technology, #3498; Bax, 1 : 1000, Cell Signaling Technology, #2772; caspase-9, 1 : 1000, Cell Signaling Technology, #9504; c-IAP, 1 : 1000, Cell Signaling Technology, #4952). The membranes were then washed with PBST containing 0.1% Tween. After three washes in PBST, each blot was incubated with peroxidase-conjugated secondary antibody for 1 h at 37°C. Labeled proteins were visualized using the Odyssey infrared scanner (LI-COR, Lincoln, NB, USA) [48]. Signals were densitometrically assessed and normalized to the *β*-actin signals, and an enhanced chemiluminescence detection system (Amersham, Piscataway, NJ, USA) was used to visualize the antibody-specific proteins in accordance with the manufacturer's recommended protocol [49].

### 2.8. Reverse Transcription-Quantitative Polymerase Chain Reaction (RT-qPCR)

Total RNA was isolated from samples according to miRNeasy Mini Kit (217004, Qiagen Company, Hilden, Germany) instructions [50]. All primers were synthesized by Takara Holdings Inc., Kyoto, Japan. RNA was then reverse transcribed into cDNA using the PrimeScript RT kit (RR036A, Takara). Next, fluorescence quantitative PCR was conducted using the SYBR® Premix ExTaq™ II kit (RR820A, Takara) on an ABI 7500 quantitative PCR instrument (7500, ABI Company, Oyster Bay, N.Y., USA). All samples were normalized to U6 and GAPDH using the 2^- *ΔΔ*CT^ method [51].

### 2.9. Mitochondrial Respiratory Chain Complex Activity Analysis

Mitochondrial respiratory chain activity was assessed using the Mitochondrial Respiratory Chain Complex Activity Assay Kit (Solarbio, Beijing, China) according to the manufacturer's instructions [52]. Briefly, the mitochondrial complex was extracted from cells and 10 *μ*l of the extract was added to each well of a 96-well plate. Detection reagents were then added to the wells followed by gentle mixing and incubation at 37°C for 2 min. Absorbance values were measured before and after the reaction using a microplate reader (BioTek, Vermont, VT), and the difference was calculated [53]. Respiratory complex enzyme activity was then calculated using the formula provided in the kit manual [54].

### 2.10. Measurement of ATP Levels

ATP production was measured using the luminometric ATP Assay kit (AAT Bioquest, Sunnyvale, CA) according to the manufacturer's instructions [55]. Briefly, H9C2 cells were seeded in a 96-well white plate and 200 *μ*l ATP assay solution was added. After mixing gently and incubating for 20 min at room temperature, luminescence intensity was measured using the luminometer mode on a plate reader (Tecan, Zurich, Switzerland) [56]. The readings were normalized to the total protein content.

### 2.11. Statistical Analysis

All results were confirmed in three independent experiments, and all quantitative data are expressed as the mean ± SD. Differences in quantitative variables between two groups were analyzed using Student's *t*-test, and differences in quantitative variables for three or more groups were analyzed by one-way ANOVA. *p* < 0.05 was considered statistically significant.

## 3. Results

### 3.1. Bevacizumab Reduces Cardiomyocyte Viability and Function

After H9C2 cells were treated with low and high concentrations of bevacizumab, cell viability was measured through a CCK-8 assay. As shown in Figure 1(a), compared to the control group, bevacizumab treatment significantly reduced cardiomyocyte viability in a dose-dependent manner. Moreover, an LDH release assay, which measures levels of LDH released into the culture medium as a result of cell membrane breakage, showed that bevacizumab-treated H9C2 cells released more LDH than control cells (Figure 1(b)). Because decreased cardiomyocyte viability is strongly associated with impaired cardiomyocyte function, we next examined single-cell contraction function in primary cardiomyocytes. While the average length of primary cardiomyocytes was not affected by bevacizumab (Figures 1(c)–1(h)), peak heights and maximal shortening velocity decreased after bevacizumab treatment, suggesting that bevacizumab disturbs cardiomyocyte contraction (Figures 1(c)–1(h)). In addition, maximal relengthening velocity and time-to-peak values increased after bevacizumab treatment (Figures 1(c)–1(h)), suggesting that bevacizumab also inhibits cardiomyocyte relaxation. Together, these results indicate that bevacizumab treatment dose-dependently reduces cardiomyocyte viability and impairs cardiomyocyte contraction/relaxation index.

### 3.2. Bevacizumab Induces Cell Apoptosis

Next, we examined alterations in cardiomyocyte apoptosis after bevacizumab treatment. First, TUNEL staining was used to observe cell apoptotic rate. As shown in Figures 2(a) and 2(b), compared to the control group, bevacizumab treatment significantly increased the number of TUNEL-positive cells in a dose-dependent manner; the low concentration of bevacizumab increased cardiomyocyte apoptosis rates to ~15%, while the high concentration increased rates to ~30%. Western blots were also performed to analyze changes in proapoptotic protein levels in cardiomyocytes. As shown in Figures 2(c)–2(e), compared to the control group, Bax, Bad, and caspase-9 protein levels increased dramatically in response to bevacizumab treatment in a dose-dependent manner (Figures 2(c)–2(e)). In contrast, Bcl-2 and c-IAP1 levels decreased significantly after bevacizumab treatment in a dose-dependent manner (Figures 2(f)–2(h)). Together, these results indicate that bevacizumab induces cardiomyocyte apoptosis.

### 3.3. Bevacizumab Treatment Is Associated with Mitochondrial Dysfunction

Mitochondrial dysfunction is considered the primary mechanism underlying chemotherapy-mediated myocardial injury. The subsequent experiments were therefore performed to analyze the effects of bevacizumab on mitochondrial function. Mitochondrial metabolism was examined first due to the importance of ATP production for cardiomyocyte viability and function. Bevacizumab treatment significantly decreased ATP production in a dose-dependent manner (Figure 3(a)). Reduced mitochondrial ATP production can result from oxidative stress and respiration dysfunction. A mitochondrial ROS probe was therefore used to analyze changes in mitochondrial oxidative stress. As shown in Figures 3(b) and 3(c), compared to the control group, mitochondrial ROS levels were significantly increased after bevacizumab treatment in a dose-dependent manner. In contrast, concentrations of antioxidative enzymes such as GSH and SOD were significantly lower after bevacizumab treatment (Figures 3(d) and 3(e)), confirming increased oxidative stress within mitochondria. In addition to mitochondrial oxidative stress, an ELISA assay also demonstrated that mitochondrial respiration complex activity (including COX-I and COX-III) decreased significantly in cardiomyocytes treated with bevacizumab (Figures 3(f) and 3(g)). These findings indicate that bevacizumab induces mitochondrial dysfunction characterized by ROS production, respiration impairments, and reduced metabolism in cardiomyocytes.

### 3.4. Bevacizumab Treatment Induces ER Stress in Cardiomyocytes

Next, we examined alterations in ER stress in cardiomyocytes treated with bevacizumab. ER stress is associated with intracellular calcium overload. An immunofluorescence assay was therefore used to examine alterations in intracellular calcium concentration. As shown in Figures 4(a) and 4(b), compared to the control group, bevacizumab treatment significantly increased intracellular calcium concentration in a dose-dependent manner. Abnormal calcium signaling activates ER stress, which is characterized by increased expression of CHOP and PERK. qPCR demonstrated that CHOP and PERK expression increased significantly in response to bevacizumab treatment (Figures 4(c) and 4(d)), indicative of ER stress activation. Excessive ER damage activates caspase-12, an upstream activator of caspase-3. An ELISA showed that caspase-12 activity increased dramatically after bevacizumab treatment in a dose-dependent manner (Figure 4(e)). Taken together, these results demonstrate that bevacizumab can induce ER stress in cardiomyocytes.

### 3.5. Bevacizumab Inactivates the ERK Pathway in Cardiomyocytes

The ERK pathway, a classical signaling pathway responsible for cardiomyocyte survival, is a potential target of many chemotherapy drugs. We therefore examined whether ERK pathway activity was affected by bevacizumab. Western blots demonstrated that the ERK pathway was inactivated, as indicated by decreased ERK phosphorylation, in cardiomyocytes after bevacizumab treatment (Figures 5(a) and 5(b)). These results demonstrated that the ERK pathway was a downstream target of bevacizumab. To understand whether ERK inactivation contributed to bevacizumab-induced cardiomyocyte death and mitochondrial dysfunction, cardiomyocytes were incubated with an ERK inhibitor (PD98059). Cell viability was measured using an CCK-8 assay, and mitochondrial function was examined by measuring ATP production. As shown in Figure 5(c), compared to the control group, PD98059 treatment significantly reduced cardiomyocyte viability, and this effect was accompanied by a drop in mitochondrial ATP production (Figure 5(d)). This finding confirmed that ERK inhibition plays a role in cardiomyocyte damage associated with bevacizumab treatment.

## 4. Discussion

The cardiotoxic effects of chemotherapy have been well documented. Although chemotherapy and immunotherapy improve the prognoses of lung cancer patients, these treatments also significantly increase the risk of myocardial injury and heart failure. In the present study, we found that bevacizumab treatment induces cardiomyocyte damage as indicated by decreased cell viability, impaired contraction/relaxation, attenuated ATP production, elevated mitochondrial ROS production, decreased mitochondrial respiration complex transcription, increased intracellular calcium concentration, and activation of ER stress. These alterations are similar to pathological changes observed in various cardiovascular disorders such as myocardial infarction, heart failure, diabetic cardiomyopathy, and hypertension, suggesting that common molecular mechanisms and signaling pathways may be involved. Furthermore, we found that the ERK pathway is inactivated by bevacizumab, and decreased ERK activity promotes cardiomyocyte death and mitochondrial damage. Overall, this study helps to explain the intracellular molecular mechanisms, including mitochondrial dysfunction, ER stress, and inhibition of the ERK pathway, that underlie bevacizumab-induced cardiovascular toxicity.

Mitochondrial damage has been proposed as the primary cause of cardiomyocyte death and dysfunction [57]. Induction of mitochondrial fission promotes cardiomyocyte death by activating the caspase-9-related mitochondrial apoptotic pathway [58]. Additionally, inhibition of mitophagy leads to the accumulation of damaged mitochondria [59]. Chemotherapy drugs also contribute to cardiomyocyte dysfunction and death by affecting mitochondrial function. For example, doxorubicin-induced upregulation of p53 inhibits protective mechanisms in cardiac fibroblast mitochondria [20], and administration of mitochondria-associated protein LRPPRC protects against doxorubicin-induced cardiac injury by inhibiting ROS production [60]. Anthracycline-mediated cardiotoxicity is also associated with dysregulation of mitochondrial metabolism, although the detailed molecular mechanisms involved are not fully understood [23]. In the present study, bevacizumab treatment resulted in mitochondrial injury associated with metabolic dysregulation in cardiomyocytes. As far as we know, this is the first study to explore the influence of bevacizumab on mitochondrial homeostasis. While recent studies have examined the relationship between morphological alterations in mitochondria and chemotherapy-induced cardiovascular damage, additional studies are required to determine whether bevacizumab also alters mitochondrial morphology.

ER stress can act as an adaptive response in cardiomyocytes [61]. Mild ER stress is characterized by increased intracellular calcium levels, which accelerate calcium-dependent ATP metabolism [62]. However, excessive ER stress is associated with the activation of CHOP and PERK, transcription factors that promote expression of apoptosis-related genes such as Bax and Bad [63]. Irreversible ER stress promotes the activation of caspase-12, which in turn directly induces caspase-3 cleavage that ultimately leads to cell apoptosis [64]. ER stress has also been identified as a potential intracellular signaling transduction mechanism underlying cardiotoxicity associated with chemotherapy drugs [65, 66]. In the present study, we found that bevacizumab treatment is associated with intracellular calcium overload, ER stress, and caspase-12 activation, suggesting that ER stress contributes to bevacizumab-mediated cardiomyocyte damage. Notably, while our data do not establish a causal relationship between ER stress and mitochondrial dysfunction, many studies have reported that ER stress may contribute to mitochondrial damage [67]. We also did not explore the possibility of interactive effects between ER stress and mitochondrial dysfunction.

Taken together, our results demonstrate that bevacizumab-mediated myocardial injury is associated with mitochondrial damage, ER stress, and ERK pathway inactivation. However, some limitations of this study should be considered when interpreting these results. First, only *in vitro* experiments were performed, and *in vivo* studies are needed to confirm our findings on the cardiotoxic effects of bevacizumab. Second, although we found that ERK inactivation is associated with cardiomyocyte death and mitochondrial damage, it remains unclear whether bevacizumab induces mitochondrial damage and ER stress specifically by directly inhibiting the ERK pathway. Third, additional bevacizumab concentrations beyond those tested here may have different effects on cardiomyocyte viability and function, and further study is needed to determine the dose threshold beyond which bevacizumab triggers cardiomyocyte damage.

## Figures and Tables

**Figure 1:** Bevacizumab reduces cardiomyocyte viability and function. (a) Cell viability was determined using a CCK-8 assay. (b) An LDH release assay was performed to examine whether bevacizumab induced cardiomyocyte damage. (c–h) The following single cardiomyocyte contractile properties were measured: peak height, maximal shortening velocity, maximal relengthening velocity, and time-to-peak. ^∗^*p* < 0.05.

**Figure 2:** Bevacizumab induces cell apoptosis. (a, b) TUNEL staining was used to observe cell apoptosis. (c–h) Western blots were used to analyze alterations in expression of apoptosis-related proteins such as Bax, Bad, caspase-9, Bcl-2, and c-IAP1. ^∗^*p* < 0.05.

**Figure 3:** Bevacizumab treatment is associated with mitochondrial dysfunction. (a) ATP production was measured via ELISA in cardiomyocytes treated with bevacizumab. (b, c) Immunofluorescence staining was used to quantify mitochondrial ROS levels. (d, e) Changes in GSH, SOD, and GPX levels were analyzed in an ELISA. (f, g) Mitochondrial respiration complex activity was examined in an ELISA. ^∗^*p* < 0.05.

**Figure 4:** Bevacizumab treatment induces ER stress in cardiomyocytes. (a, b) Intracellular calcium levels were measured using immunofluorescence. (c, d) qPCR was used to analyze changes in CHOP and PERK levels. (e) ELISA was used to detect changes in caspase-12 activity. ^∗^*p* < 0.05.

**Figure 5:** The ERK pathway is inactivated in cardiomyocytes treated with bevacizumab. (a, b) Western blots were used to analyze changes in ERK phosphorylation. (c) Cell viability was measured in a CCK-8 assay. Cardiomyocytes were treated with PD98059 to inhibit ERK activity. (d) ATP production was measured using an ELISA after PD98059 treatment. ^∗^*p* < 0.05.

## Data Availability

The analyzed datasets that were generated during the study are available from the corresponding author upon reasonable request.
